# A Structural Design of a Child Seat Based on Morphological Elements and Ergonomics

**DOI:** 10.1155/2022/1792965

**Published:** 2022-06-06

**Authors:** Xiaoshuo Jiang, Xiangjia Meng

**Affiliations:** ^1^School of Culture and Communication, Shandong Youth University of Political Science, Jinan, Shandong 250103, China; ^2^School of Information Engineering, Shandong Youth University of Political Science, Jinan, Shandong 250103, China

## Abstract

In order to improve the safety and comfort of child seat structural design, this paper combines ergonomics and morphological elements to analyze the structural design of child seat and establish a crash model. Moreover, the obtained kinematic response and injury curves are compared with the corresponding actual tested kinematic response and injury parameters to analyze the biomechanics of child occupant injury, the injury characteristics of child occupants in frontal and side collisions, and the evaluation criteria for head, neck, and chest injuries. In addition, this paper combines the intelligent design method to design a safety seat that meets the needs of children. The results show that the structural design method of child seat based on morphological elements and ergonomics proposed in this paper can play an important role in the design of child seat.

## 1. Introduction

The child restraint system is mainly designed for children, focusing on protecting the safety of children in the car, mainly composed of restraint belts, riding devices, connecting devices, fixing devices, and other auxiliary devices. The child restraint system is fixed on the inner seat of the car to reduce the injury of the child occupant by restricting the movement of the child's body in the event of a collision and ensure the safety of the child. The general car child restraint system is adjustable to meet the use of children of different ages. Child safety seat is one of the most common child restraint systems, and it is also the most used and effective child restraint system at present. It is fixed on the car seat through a connecting device and can be taken out from the car seat when not in use so as not to hinder the normal use of the car seat. In the case of the correct use of child safety seats, children's fatal injuries can be reduced by 71%, and serious injuries can be reduced by 67%. Moreover, child restraint systems play a vital role in the safety and protection of child occupants.

In the driving safety protection device, the car seat belt is designed for adults as a traditional safety protection device. However, the physical condition of children is not in line with the use of adult safety belts to protect the child's occupants from bodily injury, so it will not have a protective effect but will cause harm to the child's occupants [1]. The bones of child occupants are not as strong as adults. In the event of a car accident, the body will move forward due to the huge inertial force. At this time, the car seat belt will cause fractures, suffocation, or even breakage of children's chest ribs [2]. Car airbags are also for the protection of adults in the event of an accident. The force generated by the automatic inflation and expansion of the airbag must be fatal to younger children. There are no advantages and disadvantages, and children cannot bear this kind of force. Child safety seats are specially designed to protect children's driving safety. The correct use of qualified child safety seats that meet regulatory standards and quality assurance is the most effective way to ensure the safety of children in the car [3].

The current status of child safety seats is not optimistic, mainly in two aspects: low usage rate and high misuse rate. According to relevant surveys, although many parents expressed that they are very concerned about the safety of children in the car and intend to use child safety seats, the correct use rate of child safety seats is still not high.

The research and design of child safety seats have been relatively complete, but due to high price, inconvenient use, and complicated operation, the use rate is very low and the misuse rate is high. In order to solve the current problems in the use of child safety seats, many research institutions and automobile companies have begun to develop integrated child safety seats, also known as built-in child safety seats, which will integrate a simplified version of child safety seats into car seats. When a child is riding, the integrated child safety seat is opened and hidden when not in use so as not to affect the normal riding of adults.

This paper combines ergonomics and morphological elements to analyze the structure design of the child seat and combines the intelligent design method to design a safety seat that meets the needs of children and improves the scientificity of the structure of the child seat.

## 2. Related Work

Experiments have shown that the number of casualties caused by children under the age of 6 using child safety seats is only 1/3 of those who use safety measures in the car, so relevant parties believe that using child safety seats is the best way to protect the safety of child occupants. [4]. The importance of installing child safety seats in motor vehicles is expounded, which is a safety device to protect child occupants in the event of traffic accidents [5]. The use of child safety seats in Australia was analyzed in detail, and it was found that there were many misoperations of child safety seats, and there were also incidents that child safety seats could not be installed correctly [6]. The article proposes to enhance the safety awareness of parents and try to avoid accidents caused by the wrong operation of child safety seats. The use of child restraint systems in seven states in the United States was investigated, and the operation of the LATCH system was investigated and analyzed. The article details the critical role of the correct installation and use of car child safety seats [7]. Reports show that children who use child safety seats in a traffic accident are significantly less likely to die than those who do not [8]. Child safety seats can guarantee the safety of child occupants to a great extent [9]. Through the statistical analysis of traffic accidents, the safety test of car child safety seats and the research on the injury and protection of child occupants in traffic accidents are carried out by computer simulation experiments [10]. Several key points of research on protecting children's safety in cars are as follows: car child safety seats; the shape, internal structure, dummy simulation crash experiment; crash safety risk assessment and computer 3D modeling research [11].

Obtain the coordinate information of human skeleton nodes and the angles between key skeleton nodes through the Kinect interactive device. With the help of processing development language, Jackson realized the visualization of human movement process and the real-time transmission of data. And for designer users, real-time statistical analysis and visualization are realized [12]. The categories of existing sitting posture detection algorithms and their advantages and disadvantages are analyzed in detail. With the help of PEO sitting posture model, a nonimmersive sitting posture detection algorithm based on Kinect device is proposed. Design and implement a healthy sitting posture persuasion system and application based on human cognitive model and verify its feasibility [13]. Based on Kinect sensor, the realization method of somatosensory electronic photo album is expounded. The Kinect sensor is used to capture the human skeleton nodes, and the three-dimensional space coordinate transformation of human gestures is matched with the preset gesture library information, and then the legitimacy of the gesture information is judged and fed back to the electronic album software to complete the output instructions [14].

A seat belt and booster pad were developed for the direction to develop an integrated child booster seat cushion; for the rear child occupants under the age of 4, the seat cushion is integrated on the vehicle and is a part of the rear seat. The design also takes into account the use of seat belts. When the booster seat cushion is not used, the seat cushion can be easily restored to the seat of the adult passenger [15]. Each integrated booster seat has two levels of height adjustment to better provide comfortable restraint for children aged 4–12. This integrated booster pad is very easy to use and has a low rate of misuse, showing the importance of continuing to promote the use of child restraint systems in China [16]. The children's performance while riding in a vehicle was also studied. During the ride, children often do not sit on the seat in the correct posture due to their own wishes and the influence of vehicle dynamics. This type of research will provide a design basis for future restraint systems [17].

The influence of multipoint seat belts on child protection is analyzed by finite element simulation and trolley crash test. The results show that six-point seat belts have the best protection effect. At the same time, it is also proposed that finite element simulation analysis can replace some trolley crash tests, thereby reducing development cost and shortening the development cycle [17]. The injury status of child occupants under correct and incorrect use of child seats was studied [18]. Three kinds of crash conditions were simulated and analyzed for the integrated safety seat, and the variable design parameters were optimized [19].

## 3. A Structural Design of a Child Seat Based on Morphological Elements and Ergonomics

This article is mainly based on the latest European CRS regulation, UN ECE R129, which quantitatively analyzes the injury of the child occupant during the dynamic loading process specified in R129 by evaluating the injury parameters of the child occupant's head, neck, and chest.

According to the results of the experiment, volunteer experiment and animal experiment, the Wayne State tolerance curve, which represents the relationship between head translation acceleration, duration, and injury, is drawn, as shown in Figure 1.

In order to make the Wayne State curve suitable for various head acceleration waveforms, Versace uses the average acceleration a between any time *t*1 and *t*2 (*t*1 < *t*2) to define the head injury index (HIC):

(1) $$\begin{array}{c} HIC={\left\{\left(t_{2}-t_{1}\right){\left[\frac{1}{t_{2}-t_{1}}\int_{t_{1}}^{t_{2}}\left(\frac{a\left(t\right)}{g}dt\right)\right]}^{2.5}\right\}}_{\text{max}}. \end{array}$$

Figure 2 shows the theoretical diagram of the head injury index (HIC) using the three-axis composite acceleration waveform of the head. It corresponds to a certain time *t*_1_ of the three-axis composite acceleration so that *t*_2_ changes within the measured minimum time interval of *t*_2_ − *t*_1_ to the maximum time interval (15 ms or 36 ms). The maximum value of $\left(t_{2}-t_{1}\right)\;{\bar{a}}^{2.5}$ is sought ($\bar{a}$ is the average acceleration between *t*_1_ and *t*_2_).

In the ECE R129 regulations, the 3 ms continuous cumulative composite acceleration of the head (80 g) and the HPC^*∗*^(15) value (800) are used as the head injury evaluation indicators for 3-year-old children in the process of frontal collision.

In the ECE R129 regulations, the damage evaluation indicators for the neck of the child occupant include the upper neck axial force *F*_*z*_ and the upper neck bending moment *M*_*y*_, but they are only used for monitoring, and no damage threshold is given. The FMVSS 208 regulations stipulate that the neck damage benchmark *N*_*ij*_ is composed of the axial force *F*_*z*_ measured at the pillow and the bending moment *M*_*y*_, and the damage threshold is *N*_*ij*_ ≤ 1, and the calculation formula is as follows:

(2) $$\begin{array}{c} N_{ij}=\frac{F_{Z}}{F_{\mathrm{int}}}+\frac{M_{y}}{M_{\mathrm{int}}}. \end{array}$$

In the formula, *F*_*Z*_ is axial force; *M*_*y*_ is bending moment in buckling/extension; and subscript “int” refers to the “intercept” where the load and moment, respectively, intersect the axis.

The chest composite acceleration (duration 3 ms) is used as the damage benchmark for children's chest in UN ECE R129 regulations, and its damage threshold is 55 g. In addition, the most commonly used chest injury benchmarks include chest deformation (the displacement of the sternum relative to the thoracic vertebra) and the viscosity criterion VC value. The amount of chest deformation is highly correlated with chest injuries caused by compression, such as thoracic fractures or lung injuries. The viscosity criterion VC value is obtained from *V*(*t*) and *C*(*t*). The specific method is shown in formula (3). It is mainly to evaluate the viscous damage of the internal organs of the chest during high-speed impact from the perspective of viscous performance. The applicable range (between 3 m/s and 30 m/s) is shown in Figure 3. The resultant thoracic acceleration was measured at the fourth thoracic vertebra, T4. This injury benchmark is less relevant to injury than thoracic deformation, but since the neck, lumbar spine, shoulder joints, and restraints all transmit forces to the thoracic spine, the proportion of these forces can be studied with this injury benchmark.

(3) $$\begin{array}{c} VC=V\left(t\right)\times C\left(t\right)\\ =\frac{d\left[D\left(t\right)\right]}{dt}\times \frac{D\left(t\right)}{b}. \end{array}$$

In the formula, *V*(*t*)[*m*/*s*] is obtained by the differential of the chest deformation *D*(*t*); *C*(*t*) is instantaneous compression, that is, the ratio of the deformation *D*(*t*) at that moment to the initial breast thickness *b*. Its damage tolerance limit is *VC*_max_ ≤ 1.0m/s.

The finite element simulation software LS-Dyna was developed by Livermore Software Technologies, initially primarily to provide analysis for weapon design. LS-Dyna is a solver, and its preprocessing software includes HyperMesh, Ansys, and Patran. In the preprocessing software, the 3D model is converted into the mode of elements and nodes, and loads, constraints, and boundary conditions are applied to the finite element model, and the finally exported calculation file is the keyword file. LA-DYNA is mainly based on the Lagrange algorithm, which discretizes the continuum and mainly solves physical problems, such as explosion, collision, fluid, fluid-solid coupling, metal processing and forming, and glass forming. LS-Dyna has powerful finite element analysis capabilities and high calculation accuracy, which can accurately reflect the deformation characteristics and stress and strain of each component in the collision system, so as to provide a basis for the improvement of the model structure. The disadvantage is that due to the large number of units in the model, the modeling is complex and the calculation time is long.

Lagrange is used to describe the motion-deformation relationship of the part, and the central difference method is used for the calculation of the display integral. For microelements, the following equation can be obtained:

(4) $$\begin{array}{c} \int_{v}\rho {\overset{¨}{x}}_{i}\delta x_{i}dv+\int_{v}\sigma_{j}\delta x_{ij}dv-\int_{v}\rho f_{i}\delta x_{i}dv-\int_{v}t\delta x_{i}ds. \end{array}$$

In the formula, *σσ* is Cauchy stress tensor; *f*_*i*_ is body force per unit mass; *ρ* is displacement; *p* is mass density; *t*_*i*_ is surface distribution force: *σb*_1_*σb*_1_ is free frontier; and *V* is volume.

In (3), if the space domain occupied by the object under study is defined as Ω, the virtual displacement field is adopted, and the space domain is discretized by the finite element *I*, the following formula can be obtained:

(5) $$\begin{array}{c} \left[M\right]\left\{a\right\}=\left\{F_{ext}\right\}-\left\{F_{\mathrm{int}}\right\}. \end{array}$$

In the formula, [*M*] is quality matrix; {*a*} is nodal acceleration vector; and {*F*_ext_} and {*F*_int_} are the external and internal force vectors for the node.

Formula (5) can be displayed and integrated in the time domain using the central difference method, and the motion equations of its displacement and velocity can be calculated from the previous time step *t*:

(6) $$\begin{array}{c} {\overset{¨}{r}}^{n}=M^{-1}\left(F^{Ext}-F^{Int}\right),\\ {\dot{r}}^{n+1/2}={\dot{r}}^{n-1/2}+{\overset{¨}{r}}^{n}\Delta t^{n},\\ r^{n+1}=r^{a}+{\dot{r}}^{n+1/2}\Delta t^{n+1/2}. \end{array}$$

In the formula, Δ*t*^*n*^ is the time step at time *n*, and

(7) $$\begin{array}{c} \Delta t^{n+1/2}=\frac{\Delta t^{n}+\Delta t^{n+1}}{2}. \end{array}$$

Taking the overall displacement calculated by formula (9) and the initial position coordinates of a node as a vector operation, the coordinate data of the node at any new moment can be obtained:

(8) $$\begin{array}{c} \chi^{n+1}=\chi^{0}+r^{n+1}. \end{array}$$

The above operation steps are performed in a loop, and the time step depends on the size of the mesh and the material parameters.

The finite element model of the trolley seat in this paper is established in accordance with the dimensions and material properties specified in the UN ECE R129 regulations (as shown in Figure 4). The actual trolley seat also includes a trolley structure supporting the ECE seat and a portion of the rails connected to the trolley. This paper simplifies the trolley model and only retains the ECE seat structure, which is mainly composed of seat cushion and backrest.  Figure 5 is a three-dimensional structural diagram of the E-seat stipulated by regulations. This geometric model is preprocessed and meshed in HyperMesh 11.0, and the seat cushion and backrest geometric models are divided into hexahedral meshes and given foam materials. Since this model is a simplified model, in order to better restore the actual structure, the hexahedral mesh is covered with a layer of shell elements of rigid material.

This paper mainly analyzes the child safety seats of the front body protection type and the five-point harness type, and the test models are mainly obtained through online shopping. The front body seat is suitable for babies aged 9 months to 12 years, and the five-point carrier seat is suitable for babies aged 0–4. Its physical map is shown in Figure 6.

The geometric model of the child safety seat is obtained by reverse scanning, and the process is mainly divided into three stages, namely, data acquisition, data postprocessing, and rapid prototyping.

This article first disassembles the child safety seat purchased online and divides the disassembled parts into two parts: simple standard shape and complex shape. Simple standard shape parts are modeled in UG by hand measurement. For parts with complex shapes, such as seat frame, seat base, headrest, and so on, general 3D design software cannot accurately restore the geometric model, and these complex parts are obtained by reverse 3D scanning. The general process is as follows. The disassembled darker parts are sprayed with developer for easy scanning and identification. The coordinate points are pasted on the parts to facilitate the positioning of the parts by the instrument, and more can be pasted in places with complex structures. Next, every part of each part is scanned in as much detail as possible to obtain point cloud data for the part. It was processed into the CAD geometric model we needed using Geomagic Studio. Finally, UG is used to complete the assembly.

The postprocessing process using the reverse software Geomagic Studio mainly includes point cloud and polygon data processing, surface reconstruction and model error detection, fine modification, and assembly in UG. The general processing flow of Geomagic Studio is shown in Figure 7.

According to the above reverse scanning process, the two child safety seats mainly analyzed in this paper are disassembled and scanned. Except for the structure and shape, the reverse scanning process of the two seats is similar.

According to the 3D digital model obtained by reverse scanning, geometric cleaning and meshing were carried out in HyperMesh 11.0 to establish the finite element model of the child safety seat. The seat is mainly composed of frame, headrest, base, and other load-bearing parts, headrest with cushioning effect, flank foam, front guard board with restraint effect, and five-point harness. Other accessories, such as cloth cover, sponge, and so on, are not important structural parts, and these parts are ignored during simulation. In addition, due to the particularity of the five-point strap material, the establishment of its finite element model will be introduced in the next section.

Before using the HyperMesh 11.0 software for finite element meshing, the imported 3D digital model is geometrically cleaned, duplicate surfaces are deleted, missing surfaces are added, and some boundary lines are processed. Then, it is necessary to strictly control the grid quality standard when dividing the mesh to ensure the accuracy of the model. In the process of dividing the mesh, some noncritical parts can be simplified appropriately.

The frame, headrest, base, and other load-bearing parts of the child safety seat are divided by shell elements, and the material library of LS-DYNA software is given to MAT-24 piecewise linear elastic-plastic material (PP plastic). Among them, the base of the front body-protecting seat is made of blow molding, so the material is given to MAT-3 elastic-plastic material in the material library of LS-DYNA software. In the simulation, the real stress-strain curve is given to the material, and the real stress-strain curve is the *F* (force)-*S* (displacement) curve of the material obtained through the material tensile test.

(9) $$\begin{array}{c} \text{Nominal stress }\sigma_{e}=\frac{F}{S},\\ \text{Nominal strain }\varepsilon_{e}=\frac{\Delta l}{l},\\ \text{True stress }\sigma_{t}=\sigma_{t}\left(1+\varepsilon_{e}\right),\\ \text{True strain }\varepsilon_{t}=\ln\left(1+\varepsilon_{e}\right). \end{array}$$

Compared with conventional car child safety seats, this design simultaneously solves the problems of child riding comfort, compatibility, and safety. Compared with the prior art, the two-way riding integrated child safety seat has the following advantages. (1) It integrates two riding modes: backward and forward. The realization of backward integration can better protect the riding safety of young children so that it is suitable for a wider range of children. (2) It integrates the foldable child safety seat on the backrest of the adult seat, and the seat will not have a large displacement in the event of a collision, which is more conducive to the protection of children. In particular, when riding in a rear-facing position, children can be well protected in both frontal and side collisions due to the protection of the adult seat backrest. (3) The child rides directly on the child safety seat instead of the adult seat, so the riding comfort is greatly improved compared with the previous integrated child safety seat. (4) The foldable child safety seat can be removed from the seat back if it is not used for a long time so as not to affect the normal use of the trunk, and the folded size is small, lightweight, and easy to carry and store. (5) You can choose a five-point seat belt or a three-point seat belt to restrain the child. For infants in rear-facing and forward-facing younger children, five-point seat belts can be used for restraint while riding. For older children, three-point seat belt restraints can be used when riding forward.

## 4. Finite Element Modeling and Simulation

In this paper, the simulation analysis method of finite element-multi-rigid-body coupling is selected, and the coupling simulation model is established. According to the European regulation ECE R129, the *Q* series multi-rigid-body child dummy model is selected. The finite element-multi-rigid-body coupling analysis method is a combination of the finite element method and the multi-rigid-body system dynamics method. This coupling method is often used in the analysis of vehicle side impact. In the side impact, the response of the dummy and the deformation of the body form a coupling process of mutual influence. There are many analytical calculation methods in frontal collision simulation analysis, but sometimes they are not applicable in side collision conditions. The LS-DYNA and MADYMO coupled simulation analysis method combines the advantages of the DYNA vehicle structure finite element analysis and the NADYMO multi-rigid dummy restraint system analysis. This coupling calculation not only avoids the situation that the calculation is terminated due to the negative volume that often occurs in the calculation process, but also can quickly reflect the occupant injury situation, and is suitable for side impact and frontal impact simulation analysis. The principle of coupling analysis is that the LS-DYNA and MADYMO conduct coupling analysis through a coupling interface, and information from one software to another is carried out through the same coupling interface. The solvers of the two software operate at the same time, complete the transfer and exchange of data in the process of operation, and obtain the required data, respectively.

In this study, the structural deformation of the child safety seat needs to be considered, and at the same time, the injury and movement of the child occupant during the crash simulation process should be analyzed. In addition, children's models of multiple age groups need to be used, so the multi-rigid-finite element coupling analysis method can not only meet the requirements of result analysis, but also reduce the workload and speed up the calculation speed. The collision simulation coupling model is established through the coupling interface. In the end, not only the structural deformation of the child safety seat can be well responded, but also the damage value and movement of the child dummy can be well responded. The steps for establishing the coupling model in this paper are as follows:

(1) The three-dimensional model of the seat is imported into the HyperMesh software, and the finite element model of the seat was established, including two models of forward and backward. (2) Multi-rigid child dummies of different age groups are selected, and a five-point seat belt restraint system is established in MADYMO software. (3) The seat finite element model and the child-safety belt multi-rigid body model were imported into the Coupling Assistant software for coupling, the sitting position of the child dummy was adjusted, and the contact between the finite element model and the multi-rigid body dummy was established. (4) The coupled model is derived and the results are calculated. The specific flowchart is shown in Figure 8.

On this basis, the effect of the structural design method of the child seat based on morphological elements and ergonomics proposed in this paper is verified, and the evaluation score of the structural effect of the child seat designed in this paper is calculated. This paper mainly evaluates from two perspectives of safety and comfort, and the results shown in Tables 1 and 2 are obtained.

From the above research, it can be seen that the design method of the child seat structure based on morphological elements and ergonomics proposed in this paper can play an important role in the design of child seats.

## 5. Conclusion

In order to increase the popularity of child safety seats, improve the quality of child safety seats, increase the safety of child safety seats, and reduce children's sense of restraint on the seat, this paper analyzes and summarizes the shortcomings of existing car child safety seats through the analysis of children's physiology and psychology. Moreover, this paper conducts a survey on the design requirements of child safety seats for existing users and better integrates user needs into the design of intelligent child safety seats to provide children with both physical and psychological protection. This paper combines ergonomics and morphological elements to analyze the structural design of the child seat and combines the intelligent design method to design a safety seat that meets the needs of children. The results show that the structural design method of child seat based on morphological elements and ergonomics proposed in this paper can play an important role in the design of child seat.

## Figures and Tables

**Figure 1:** Wayne State tolerance curve.

**Figure 2:** HIC solution process.

**Figure 3:** Scope of application of the viscosity criterion.

**Figure 4:** 3D model.

**Figure 5:** Finite element simulation model.

**Figure 6:** Physical simulation of the child seat. (a) Front-guard-type CRS. (b) Strap-type CRS.

**Figure 7:** General processing flow of Geomagic Studio.

**Figure 8:** Modeling process.

**Table 1:** Safety evaluation of the design method of child seat structure based on morphological elements and ergonomics.

Num	Safety	Num	Safety	Num	Safety	Num	Safety
1	91.22	16	93.84	31	89.26	46	88.93
2	92.16	17	92.61	32	87.90	47	91.49
3	88.41	18	92.89	33	90.64	48	93.61
4	88.70	19	88.26	34	91.03	49	88.59
5	89.31	20	89.21	35	89.67	50	87.29
6	93.17	21	88.91	36	92.30	51	88.90
7	92.15	22	91.10	37	88.04	52	87.51
8	92.50	23	90.09	38	90.75	53	92.42
9	89.70	24	90.35	39	90.65	54	90.86
10	92.10	25	92.05	40	88.35	55	89.25
11	87.14	26	93.88	41	89.88	56	91.20
12	90.50	27	87.48	42	88.63	57	91.70
13	87.28	28	89.99	43	87.87	58	88.10
14	89.69	29	89.28	44	93.67	59	87.68
15	89.04	30	88.88	45	90.18	60	89.02

**Table 2:** Comfort evaluation of the design method of child seat structure based on morphological elements and ergonomics.

Num	Comfort	Num	Comfort	Num	Comfort	Num	Comfort
1	81.84	16	81.80	31	81.77	46	81.37
2	81.37	17	81.24	32	81.29	47	81.63
3	81.65	18	81.90	33	81.17	48	81.24
4	81.32	19	81.93	34	81.89	49	81.07
5	81.98	20	81.98	35	81.35	50	81.18
6	81.08	21	81.16	36	81.67	51	81.68
7	81.72	22	81.99	37	81.12	52	81.45
8	81.77	23	81.07	38	81.34	53	81.59
9	81.79	24	81.19	39	81.87	54	81.63
10	81.83	25	81.75	40	81.79	55	81.36
11	81.98	26	81.53	41	81.32	56	81.52
12	81.75	27	81.35	42	81.24	57	81.63
13	81.20	28	81.23	43	81.45	58	81.55
14	81.32	29	81.76	44	81.33	59	81.48
15	81.12	30	81.71	45	81.50	60	81.53

## Data Availability

The labeled dataset used to support the findings of this study are available from the corresponding author upon request.
